This article has been retracted.

# Economic Order Quantity Model-Based Optimized Fuzzy Nonlinear Dynamic Mathematical Schemes

**DOI:** 10.1155/2022/3881265

**Published:** 2022-07-15

**Authors:** Kalaiarasi Kalaichelvan, Nasreen Kausar, Sajida Kousar, Yeliz Karaca, Dragan Pamucar, Mohammed Abdullah Salman

**Affiliations:** ^1^PG and Research Department of Mathematics, Cauvery College for Women (Affiliated to Bharathidasan University), Tiruchirappalli 620018, Tamil Nadu, India; ^2^Department of Mathematics, Yildiz Technical University, Faculty of Arts and Science, Esenler 34210, Istanbul, Turkey; ^3^Department of Mathematics and Statistics, International Islamic University Islamabad, Islamabad, Pakistan; ^4^University of Massachusetts Medical School (UMASS), Worcester, MA 01655, USA; ^5^Department of Logistics, University of Defence in Belgrade, Belgrade, Serbia; ^6^College of Education, Applied Sciences and Arts, Amran University, Amran, Yemen

## Abstract

Fuzzy mathematics-informed methods are beneficial in cases when observations display uncertainty and volatility since it is of vital importance to make predictions about the future considering the stages of interpreting, planning, and strategy building. It is possible to realize this aim through accurate, reliable, and realistic data and information analysis, emerging from past to present time. The principal expenditures are treated as fuzzy numbers in this article, which includes a blurry categorial prototype with pattern-diverse stipulation and collapse with salvation worth. Multiple parameters such as a shortage, ordering, and degrading cost are not fixed in nature due to uncertainty in the marketplace. Obtaining an accurate estimate of such expenditures is challenging. Accordingly, in this research, we develop an adaptive and integrative economic order quantity model with a fuzzy method and present an appropriate structure to manage such uncertain parameters, boosting the inventory system's exactness, and computing efficiency. The major goal of the study was to assess a set of changes to the company current inventory processes that allowed an achievement in its inventory costs optimization and system development in optimizing inventory costs for better control and monitoring. The approach of graded mean integration is used to determine the most efficient actual solution. The evidence-based model is illustrated with the help of appropriate numerical and sensitivity analysis through the related visual graphical depictions. The proposed method in our study aims at investigating the economic order quantity (EOQ), as the optimal order quantity, which is significant in inventory management to minimize the total costs related to ordering, receiving, and holding inventory in the dynamic domains with nonlinear features of the complex dynamic and nonlinear systems as well as structures.

## 1. Introduction

The importance of nonlinear combining forecasts, which play a role in robust and accurate forecasting, needs to be investigated further. Thus, there are studies, which make use of classifiers using bevelled edges (FNN) employed as a complex integrating predictive tool. The research concluded that FNN exceeds individual predictor variables and exponential trying to combine algorithms in order to accurately predict quality. The advantage of FNN is credited to its capacity to cope with address extremely nonlinear dynamical and temporal correlations that typical simulations would adequately grasp that analyses the necessity and methodology of world trade export predicting that are described but also the underlying systems for projecting deep neural and fuzzy concept conceptions. The authors of the article used a computational model and probability logic to construct a statistical model that estimates the transition frequency of global trade commodities.

Leveraging semi features, such as blurry multivariate statistical concepts aligned against timestamps, seems to have become a significant line of science since fuzzy conventional statistical simulations would not demand rigid inference digital mainstream empirical methods that necessitate the fulfilment of some generalizations [1, 2]. As an outcome, research aims at a premium quality regression-based paradigm inside which individual possesses are properly considered and neural nets are deployed to detect fuzzy relations. Dutt et al. [3] presented approach highlights how crossover processors are also used to contend with a big combination of bits, and the scientists have used the clustering algorithm for convolution. The study provides the evaluation of forecasting performance conducted by the application of the proposed method, which shows its superior performance as supported by a related simulation that proposes a high-end rank detrended fluctuation algorithm for strengthening prediction. The investigators use a lower order imprecise multivariate statistical system based on adapted hope and neural network for this function, which is now being established to drastically improve predicted effectiveness. Some other analyses, based on multi dynamics, explore the temporal impact of lost profits or use the extensively adopted preparation policies with entity delivery times.

In parallel to the study helps to identify above, Zhang and Liao [4] initiated gathering flawed data by applying compiled code *k*-means and *k* methodology to motivate and encourage intuitionistic, and c-means encryption method central processing letters. Inventory management is the recording of assets, component aspects, and building materials being used, which are sold by an organization. As a business person, it manages inventory to assure that you have appropriate stock on hand and to identify once there is a deficiency. In budgeting, merchandise is a physical resource that typically alludes to all commodities in distinct steps of construction. If companies and factories conserve goods, they would actually sell and make products. For most organizations, inventory is a valuable consideration in the trial balance; unfortunately, holding excessive material can be a central challenge. Pham et al. [5] developed a probabilistic reasoning model, which was built for quality assurance. The cycle counting paradigm of inventory levels featuring varying customer demand is considered. The article outlines the kinematics of the power generation system in a controlled conceptual way.

Intuition is a parameter computing strategy that enables the evaluation among several distinct posterior probabilities with about the same value. Pattern recognition tried to address problems by leveraging an extended, faulty spectrum of realities and judgements that provides for a vast scope of accurate predictions to be established. To illustrate various sub of a dichotomous scale, a simple programme could well be implemented. Li et al. [6] devised a classifier algorithm based on proximity spacing for an optimization technique with limited data. A calorimeter for generally pro restraints should also include a multitude of connection weights that indicate the air temperature needed to fully operate the closures. Each device captures the same actual temperature to correctness in 0 to 1 domain. These original values could be used to understand how to use the brake pedal. The heuristic approach will be used to indicate doubt.

Fuzzy logic is vital for both researchers and practitioners because of its economical and real uses, which also include the potential to modulate manufacturing and home appliances, not supplying precise rationality but still some thinking, and designers were able to incorporate fuzzy approach to cope with ambiguity [7]. Automation (ML) is a type of neural network (AI) that enables technology initiatives to improve their generalization ability without ever being penalized to do so. Neural nets utilize existing data is fed to determine the contemporary final output. Automation delivers alternative answers from massive amounts of data by building algorithms for analysing real-time data and providing reliable findings and analysis [8]. The goal of automation is to produce digital programmes that access collections and educate on self. The fundamental benefit of ML algorithms is that once the algorithm discovers or comprehends how to analyse data, it will do so automatically. Human learning will be ineffective in cases of high data volume. Because fuzzy clustering permits genes to belong to many clusters, it can identify genes that are conditionally coregulated or coexpressed.

## 2. Materials and Methods

Maintaining and improving data quality in nonlinear dynamic models is particularly crucial for developing accurate and trustworthy planning and making smart decisions, leading to a better decision-making and a reliable precondition of such processes. This line of procedures ensures the decreasing of risk and increasing of confidence, which brings about consistency and improvements in results. It is also acknowledged that planning techniques, including the features of data quality dimensions, quality characteristics, and quality indexes, require data and expertise as well as human-computer interaction. Informatics is the study of developing a new knowledge system via the collection and categorization of data utilizing computers and networks. In order to validate the model with the actual track of the current way of operation, it has been found that the EOQ is not matching with the lot size and the replenishing quantity. Hence, reconsideration was done with respect to the actual lot size and quantity of replenishment. Traditional *K*-means clustering works well when applied to small data sets. Large data sets must be clustered such that every other entity or data point in the cluster is similar to any other entity in the same cluster.

It involves the application of computer science, information science, and some domain expertise to develop new insights and improve knowledge discovery. Informatics of resources may be regarded as a tool that allows material scientists to obtain new insights into their data by combining a variety of machine learning algorithms with novel schemes for data visualization, more interaction with data, and domain experts. It can expedite inquiry and eliminate information systems. This will be driven by massive growth in the field of information technology, which is boosting interest in the use of expert systems, knowledge discovery, pattern recognition, retrieval, semantic technology, and other smart applications.

Learning is an effective process for recognizing structure in data set. Clustering is the method of collecting groupings whereby inhabitants are associated in some way [9]. A cluster is, therefore, a group of objects or events to each other diverse from the elements in other clumps. Data clusters of reducing large statistics into smaller are of the same data. Categorization is used to spawn the taxonomic classification procedure expediently. It defines how the values of fast data are collected but also integrated.

When merged, cluster analysis or digital logic allows simple yet effective techniques for modelling difficult problems. Proposed technique offers a useful and adaptable approach to identifying masses of material elements by allowing so same data item to appear in very many clusters with various class labels. Identification categories can be described as affinity, choice, or hesitation [10]. Granular categorization will be used to evaluate how related a product or incident is to a technology demonstrator, to offer alternatives among suboptimal fixes or to reflect perplexity about the true state if it is conveyed in careful wording.

Even though vague strategies are so similar to real logic, the conclusions it delivers are easy to understand and apply. Neural nets are a suitable process for describing imprecise, equivocal, or unclear because of these properties. Other classification methods would be used although we opted for the clustering means approach, which is simple and simplistic. Thresholding is a data classifier that classifies a collection into *n* regions, for each piece of evidence in the collection and sometimes very fitting to each category. A source of data at the midst of a cluster, for example, has a considerable standard of connecting or involvement to such clusters, while a piece of evidence far off from the middle of a grouping has a slight amount of adhering to or connection with that array.

### 2.1. Economy Data Set

Sorting is a significant big data analysis information mining approach that attempts to simplify the elementary and intermediate tuples (patterns) such that items placed in almost the same region are identical and uniform focused upon such qualities. The object is to reorganize a list of images so that some in the same category are more associated with these other groups (clusters). It should be noted that deep classification should be used in clumping. If we consider each sort of signal to be a feature, we may use feature selection to discover the most important signals [11]. These signals can then be used by process engineers to identify critical elements that contribute to yield excursions downstream in the process. The data set offered in our study is a subset of those attributes, with each example representing a single production item with accompanying measured features. All costs associated with preparing a purchase order are termed as ordering costs, which include the cost of preparing a purchase invoice, telephone, salaries of purchasing clerks, and stationery. It does not include the actual cost of the goods. Data collection is the process of gathering and measuring information on targeted variables in an established system, which then enables one to answer relevant questions and evaluate outcomes. First, we clean the data by removing unnecessary variables and imputing missing values. The observed products are then divided into two subsets using the K-means clustering: one group of failed items and one group of perfect products. The cluster analysis is then applied just to the data set, which does not perform well for accurate clustering that yields the significant attributes for a successful clustering process.

### 2.2. Methodology

Clusters are allocated a membership value in fuzzy clustering. Fuzzy clustering methods enable clusters to expand. In other circumstances, the membership value is very low, suggesting that the concerned data point is not a member of the cluster under examination. Some crisp approaches have difficulty dealing with outliers; however, in the case of fuzzy procedures, these outlier points are assigned a low degree of membership. The membership degree indicates whether or not the data point is a member of a cluster. As a result, fuzzy logic is the sole way to deal with data that is ambiguous or uncertain. The fuzzy *C*-means (FCM) method incorporates operations that entail the determination of cluster centres and the assignment of points to these centres using a formula known as Euclidian distance. Automated fuzzy clustering is a clustering approach that delivers one data or picture element that belongs to two or more groups. The strategy algorithm assigns input value towards each image location attached to each centroid based on its centre of mass. Thresholding clusters is a foundation on which to build algorithm in which every parameter is handed chances or hazard brackets whether it relates to a few subgroups.

### 2.3. Economic Order Directory Management Scheme with Fuzzy Clustering

Most firms that deal with inventory management devote a significant amount of work to optimization approaches. Algorithms may be developed to match bespoke limitations that suit your business with the use of artificial intelligence and machine learning. This can help with inventory optimization, especially in companies with many distribution centres. These models can be tweaked to account for independent circumstances that may cause product delivery to be delayed [12]. Machine learning to optimize inventory space is a more effective technique of managing stock when it comes to elements impacting inventory management. The nonlinear relationships between the objective function and the decision variables, and the constraints and the parameters introduce varieties of complexities in optimization models. Last century was an era of development in the field of nonlinear modelling of real-life problems. *K*-means looks for a fixed number (*k*) of clusters in a data set. A cluster refers to a collection of data points aggregated together because of certain similarities. You shall define a target number *k*, which refers to the number of centroids you need in the data set. By devoting this effort to artificial intelligence, more attention can be paid to product quality and customer experience, resulting in improved corporate success.

In many of today's businesses, using machine learning to reduce the variables that affect inventory management has become more popular. Businesses may use it to increase stock tracking accuracy, optimize inventory storage, and provide transparent supply chain interactions, to name a few of the numerous applications [13]. In this due consideration, enhancing the reliability and effectiveness of asset tracking and management technology has provided precise information in subsequent planning and policy facility for sustainable growth.

### 2.4. Remunerative Arrangement Grouping Scheme for Indistinct Directory

The market equilibrium is the appropriate Pickering equation for an organization to collect, in order to minimize stock-outs such as collecting expenses, inadequacy prices, and procurement fees (EOQ). This performance approach was introduced by Ford W. Harris in 1913, and this has been continuously improved. Estimate, pricing, purchasing, and related costs are all held constant. These elements contain the following details:

- Demand forecasting (EOQ) is the aggregate planning frequency for a company's net issuing, shipping, and storage material charges.
- The quantity discount algorithm works when desire, supply, and overheads are all predictable with time.
- Most prominent weaknesses of the coefficient of determination are that it requires growing appetite for the latest sales across time.

The intent of the statistical model is to identify the optimal couple of new units to order. If this purpose is accomplished, a company's spending for selling, shipping, and retaining equipment can be lessened [14]. Large corporations' expenses determine to reorder point using a programme in their application, and the reorder point methodology may be tweaked to estimate multiple productions or request times.

Under today's volatile situations, expecting undiscovered variables is a vital financing strategy. Any original circumstance concern can be established and estimated as a variable of date of filing. If a definite reliability at a specific date is desirable, optimized models are able to estimate the preliminary accuracy involved to attain it. Short-term predictions of dynamical systems, on the other hand, are critical for risk assessment and delivering right info of protracted ruling mechanisms. The fractional-order nonlinear equal width models are very significant partial differential equations that identify the numerous complex nonlinear occurrences in science's research area, especially in chemical physics, thermal waves, plasma physics, solid physics, fluid mechanics, etc. Variable compensation is pay given to an employee based on the results they produce. It is usually offered on top of a fixed salary and comes in various forms. Commission: this is a portion of revenue given to the sales employee as part of an official compensation plan.

The precision of summary recommendations is dependent on the following major factors: the competence of classifiers to extrapolate effectively on heretofore unknown data and the underlying repeatability of behaviours. As a result, the approach might assist an organization in monitoring the number of dollars from its final price. Apart from assets, the most significant result is that these organizations and companies demanded resources in place to satisfy customers' expectations. If demand forecasting (EOQ) enabled you to drop your inventory system, the extra income could also be used for another identifying the skills or pledge.

### 2.5. Cluster Analysis Scheme Using Fuzzy Economy Data with Defective Module

The derived total profit is

(1) $$\begin{array}{c} TC=\frac{ka\left(\lambda -d-a\right)}{Q\left(\lambda -d\right)}+\frac{Q\left(h+\delta \mu \right)}{2}. \end{array}$$

Clustering algorithm is one of the most often used unsupervised learning approaches. They are frequently used as one of the initial steps in data analysis to offer a basic understanding of the structure of a data collection. Normalization is the task of defining a cluster of products under sections or “agglomerations” so that articles in just the same class are comparable and objects in other classes are unique. In certain cases, the purpose is to organize the clusters into a natural hierarchy (hierarchical clustering). Cluster analysis may also be used as a type of descriptive statistics, indicating the data are divided into separate groupings. Clustering methods are commonly used as input information on the (pairwise) similarity between items, such as a proximity matrix [15]. Objects are often defined in terms of a collection of measures from which similarity degrees between pairs of objects may be calculated using a similarity or distance measure. Defect clustering in practice demonstrates how defect dispersion is not widely distributed across the programme, but it is rather concentrated in a small region of the application. It is essentially a huge system in which changes in size, complexity, and errors have an influence on the system's quality and can damage a specific module.

## 3. Experimental Results and Discussion: Mixture Fuzzy Modelling with Categories of Clustering Algorithms for Economy Data

Instead, they start with a maximizing objective function and treat clustering as a combinatorial optimization issue. Mode-seekers are models that are similar to mixture models. They, on the other hand, employ a nonparametric approach and attempt to estimate modes of component density functions directly. The distance between the items and the modes that act as cluster centres is then used to build clusters. The most well-known example of this class is probably the *K*-means algorithm. The goal of *K*-means is to reduce the sum of the squared error over all clusters in line with

(2) $$\begin{array}{c} J\left(C\right)=\sum_{k=1}^{K}\sum_{x_{i}\in c_{k}}{\left\|x_{i}-\mu_{k}\right\|}^{2}. \end{array}$$

In traditional clustering, each item is categorically allocated to one of the clusters. As a result, strong borders divide the distinct clusters. Such restrictions are sometimes unnatural or even irrational in practice. Rather than being abrupt, the boundary of single clusters and the transition between various clusters are frequently smooth (see Figure 1). This is the driving force for fuzzy clustering method extensions [16]. An item can belong to many clusters at the same time in fuzzy clustering, at least to some extent, and the degree to which it belongs to a given cluster is described in consideration of level. It is commonly believed that the membership functions of the various clusters (specified on the set of observed points) form a partition of unity.

This variant, also known as probabilistic clustering, can be made broader by loosening the requirement. The *k*-means algorithm divides a given collection of observations into a predetermined number of *k* groups. Because of its efficiency, the *K*-means algorithm is a common technique [17]. Fuzzy clustering has shown to be quite beneficial in reality, and it is now widely used outside the fuzzy community. It may appear vague, but if a business begins scouring its metrics for serious issues focusing on a specific application. When testing software, testers frequently encounter situations in which the majority of the faults discovered are connected to a certain feature and the remaining capabilities have a lesser number of errors. Defect clustering refers to a limited number of modules that contain the majority of the flaws. Essentially, flaws are not dispersed consistently throughout the programme, but rather are concentrated or consolidated among two or three functionalities. Due to the intricacy of the programme, coding may be hard or tricky at times, and a developer may make a mistake that affects only a single functionality or module. As a result, if the improvement campaign focuses on a certain programme, the largest gains might be realized. Instead of overflowing everything else in the meantime, repurposing a little more resources and muscle can make a difference in the focused technology.

### 3.1. Clustering Technique Based on *K*-Means with Defective Module Based on Mixture Fuzzy Modelling for Economy Data

It is also the most elementary autonomous learning model for aggregating issues. The K-means algorithm partitions *n* events into different clusters, from each observer going to a colony, and the corresponding necessarily implies providing as a precedent.

Figure 2 shows that the k-means sorting method essentially performs two main objectives: continually discovering the average mean for K grid points or number of clusters and placing each piece of information to the *k*-centre that seems to be adjacent to it. Variables that are closer to a common *k*-centre produce a grouping.

The derived total profit is

(3) $$\begin{array}{c} TC=\frac{ka\left(\lambda -d-a\right)}{Q\left(\lambda -d\right)}+\frac{Q\left(h+\delta \mu \right)}{2}, \end{array}$$

(4) $$\begin{array}{c} \begin{array}{c} \partial J\;TC\left(Q\right)=\frac{1}{6}\left\{\left[-\frac{k_{1}a\left(\lambda -d-a\right)}{Q^{2}\left(\lambda -d\right)}+\frac{Q\left(h_{1}+\delta \mu \right)}{2}\right]+2\left[-\frac{k_{2}a\left(\lambda -d-a\right)}{Q^{2}\left(\lambda -d\right)}+\frac{Q\left(h_{2}+\delta \mu \right)}{2}\right]\right.\\ \left.+2\left[-\frac{k_{3}a\left(\lambda -d-a\right)}{Q^{2}\left(\lambda -d\right)}+\frac{Q\left(h_{3}+\delta \mu \right)}{2}\right]+\left[-\frac{k_{4}a\left(\lambda -d-a\right)}{Q^{2}\left(\lambda -d\right)}+\frac{Q\left(h_{4}+\delta \mu \right)}{2}\right]\right\} \end{array}. \end{array}$$

If we equate it to zero, then we obtain the crisp quantity.

(5) $$\begin{array}{c} Q=\sqrt{\frac{\left(\lambda -d-a\right)\left(k_{1}a+2k_{2}a+2k_{3}+k_{4}a\right)}{\left[\left(h_{1}+\delta \mu \right)+2\left(h_{2}+\delta \mu \right)+2\left(h_{3}+\delta \mu \right)+\left(h_{4}+\delta \mu \right)\right]\left(\lambda -d\right)}}. \end{array}$$

The automated classification system uses ambiguous clustering in which one set of data or images is absolutely essential to the averages of two groups. Following equation includes the entire cost of an imprecise mixed modelling blend [6]. The algorithm distributes similarity score to each individual frame associated with each cluster centre proportion to the distance between centroid and the image point. Aggregation is seen in fuzzy imagery supplied with *k*. In pattern matching, Equations 2 and 3 are used to diminish faulty items. A cluster of data sets has been placed together, so they share common qualities. It is important to first define a specific number, *k*, for the quantity of clustering requested in the set. A centre of mass is a mythical or legitimate position that defines the centroid.

(6) $$\begin{array}{c} Q_{1}=Q_{2}=\frac{2\left[k_{4}a\left(\lambda -d-a\right)\right]+4\left[k_{3}a\left(\lambda -d-a\right)\right]}{\left[h_{1}+\delta \mu +12\lambda \right]\left(\lambda -d\right)+\left[2\left(h_{2}+\delta \mu -12\lambda \right)\right]\left(\lambda -d\right)},\\ Q_{1}=Q_{2}=Q_{3}=\frac{2\left[k_{4}a\left(\lambda -d-a\right)\right]+4\left[k_{3}a\left(\lambda -d-a\right)\right]+4\left[k_{2}a\left(\lambda -d-a\right)\right]}{\left[h_{1}+\delta \mu +12\lambda \right]\left(\lambda -d\right)+\left[2\left(h_{2}+\delta \mu -12\lambda \right)\right]\left(\lambda -d\right)+2\left[h_{3}+\delta \mu -12\lambda \right]\left(\lambda -d\right)},\\ Q_{1}=\sqrt{\frac{2\left[k_{4}a\left(\lambda -d-a\right)\right]}{\left[\left(h_{1}+\delta \mu \right)+12\lambda_{1}\right]\left(\lambda -d\right)}},\\ Q_{2}=\sqrt{\frac{4\left[k_{3}a\left(\lambda -d-a\right)\right]}{\left[\left(h_{2}+\delta \mu \right)-12\lambda_{1}+12\lambda_{2}\right]\lambda -d}},\\ Q_{3}=\sqrt{\frac{4\left[k_{2}a\left(\lambda -d-a\right)\right]}{\left[2\left(h_{3}+\delta \mu \right)-12\lambda_{2}+12\lambda_{3}\right]\left(\lambda -d\right)}},\\ Q_{4}=\sqrt{\frac{2\left[k_{1}a\left(\lambda -d-a\right)\right]}{\left[\left(h_{4}+\delta \mu \right)-12\lambda_{3}\right]\left(\lambda -d\right)}}. \end{array}$$

The solution $\tilde{Q}=\left(Q_{1},Q_{2},Q_{3},Q_{4}\right)$ satisfies all inequality constraints.

(7) $$\begin{array}{c} Q^{*}=\frac{\left(\lambda -d-a\right)\left[2k_{4}a+4k_{3}a+4k_{2}a+2k_{1}a\right]}{\left(\lambda -d\right)\left[h_{1}+\delta \mu +2h_{2}+\delta \mu +2h_{3}+\delta \mu +h_{4}+\delta \mu \right]}. \end{array}$$

It requires electronically finding hidden pattern in data. For training set (including prediction), association rules basically analyse the input messages and search for spontaneous groups in classifier. The clustering algorithm is an unsupervised technique in which the input is not labelled and issue resolution is relied on the algorithm's expertise in tackling similar problems as a training schedule. While statistical randomness arises due to lack of adequate data and variability in a system, fuzziness incorporates imprecision arising from lack of complete information, conflicting viewpoints or theories, incomplete or incorrect models of physical phenomenon, and subjective decisions made during analysis. Fuzzy *c*-means clustering has can be considered a better algorithm compared to the *k*-means algorithm. Unlike the *k*-means algorithm where the data points exclusively belong to one cluster, in the case of the fuzzy *c*-means algorithm, the data point can belong to more than one cluster with a likelihood. Defect clustering occurs when flaws are not evenly spread throughout a programme, resulting in a large number of small features causing a severe quality concern.

For the goal of fault clustering, a variety of culprits are used. The veracity of every assertion becomes a question of degree in fuzzy logic [18]. Fragmenting faulty information efficiently through using *k* analysis based on cores neural component symbol categorization, generally described as trying to sort, is a technique that demands the utilization of those feature extraction. It demands the electronic investigation of concealed data sets. Connection rules actually examine the process that is the creation and looking for spontaneously subgroups in the classification for the training data set (containing predicting).

### 3.2. Fuzzy Mathematical Modelling in Defective Items Using Cluster

After the model is trained, its performance is needed to be seen. While accuracy functions give information on how well a model is functioning, they do not provide information on how to improve it. A correctional function is to be needed in order to figure out when the model is the most accurate, as there is the need to find the sweet spot between an undertrained and an overtrained model.  Figure 3 shows that a cost function of equation (4) is used to determine how inaccurate the model is in determining the relationship between input and output. It indicates how poorly the model in question is performing and forecasting.

In our study, we also demonstrated that using a succession of two separate clustering algorithms to discover and categorize errors in the manufacturing process may be an effective and successful strategy. The type and source of the data can be regarded as the constraints of this study (see Algorithm 1). The higher the similarity level, the more similar the observations are in each cluster. The lower the distance level, the closer the observations are in each cluster. Ideally, the clusters should have a relatively high similarity level and a relatively low distance level.

The data set in this example is obtained from a public source; therefore, there was very little supplemental information regarding the production environment. As a result, the quality of the data set may be viewed as a possible constraint [19]. The Firefly optimization approach is used in conjunction with the traditional fuzzy C-mean clustering technique. As a result, our proposed technique can automatically recognize the faulty picture region with more accuracy than existing defect detection methods. Convolutional neural network-based image segmentation may be utilized in the future to differentiate defective and defect-free areas in coating surfaces.

## 4. Conclusions and Future Directions

The economic order quantity (EOQ), as the optimal order quantity, is crucially important in inventory management to minimize the total costs concerned with ordering, receiving, and holding inventory. In that regard, group method is beneficial for businesses, companies, institutions, entities, and organizations attempting to identify individual customer groups, transaction data, and perhaps other type of transactions and commodities. Filtering, widely referred to as data sets, is an important file interpretation practice. It accurately uncovers categories (made reference to as groupings) in large data set, with fragments even in the same is more identical evaluation metrics. The main objective of all this study's fuzzy aspect is to separate data into groups; for each measurement, it is assigned a similarity score one per cluster. Economic order quantity (EOQ) is a calculation that companies perform to represent their ideal order size, allowing them to meet demand without overspending. Inventory managers calculate EOQ to minimize holding costs and excess inventory. Compared with the *K*-means strategy, which demands pieces of information to be allotted to just one column, the imprecise *K*-means methodology allows pieces of information to be attributed to many categories with a frequency. Fuzzy *K*-means segmentation trumps traditional methodologies for redundant time series. The classifier is used in the available data set to differentiate between products that survived checking and all those that did not. In this context, we need groupings to be able to identify between those that qualified and those that refused. The *K*-means approach has been opted for in this study since the number of clusters requires to be obtained. Following the identification of the failed product group, the hierarchical clustering approach will be utilized to investigate the location of the defect origin. Being one of the most extensively used clustering methods, *K*-means clustering is prioritized by individuals and researchers when they need to work on and sort out a clustering problem to grasp the nature, structure, and particularities of the data set in question [20].

Accordingly, this paper aims at justifying the method employed to minimize the cost function mathematically through algorithmic application. Clustering is not, in general, categorization or prediction. However, you may use the knowledge gathered through clustering to try to enhance your categorization. Simulation model estimates enable firms to achieve high precision guesses about the predicted values of a request basis of previous experience that might be about anything to do with lost business to possible misrepresentation. Machine learning approaches for decision-making generate accurate outcomes while dealing with massive data environments and provide valuable suggestions to specialists in many industries for future upgrades in the sectors in which they are involved. Fuzzy logic also aids in determining the uncertainties in an issue, adapting to changing settings and assisting in decision-making. The reviewer performance in this study provides an idea that machine learning is a developing subject with spur than fuzzy logic [21]. Considering these aspects, fuzzy mathematics-informed methods prove to provide benefits in conditions when observations show uncertainty and volatility. Therefore, it becomes vital importance to make predictions about the future considering the stages of interpreting, planning, and strategy building. It is possible to realize this aim through reliable, accurate, and realistic data and information analysis, emerging from past to present time. As a result, to increase the performance of fuzzy logic, we may improve the fuzzy extensions on other algorithms as future research content. Therefore, the present study has had the aim of pointing a new direction, considering EOQ as the optimal order quantity, which is significant in inventory management to minimize the total costs concerned with ordering, receiving, and holding inventory in the ever-changing dynamic fields with regard to the complex dynamic and nonlinear systems as well as structures.

## Figures and Tables

**Figure 1:** Clustering algorithms for economy data based on mixture fuzzy modelling.

**Figure 2:** Clustering technique in *K*-means based on mixture fuzzy modelling for economy data.

**Figure 3:** The defective items detected in economy data.

**Algorithm 1:** Fuzzy mathematical model algorithm.

## Data Availability

No data are used to support this study.
